# Value Proposition for Enabling Construction Project Innovation by Applying Building Information Modeling

This article has been retracted.

**DOI:** 10.1155/2022/2586307

**Published:** 2022-01-07

**Authors:** Hui Liu, Qianqian Ju, Na Zhao, Hujun Li, Miroslaw J. Skibniewski

**Affiliations:** ^1^Department of Engineering Management, School of Management and Engineering, Zhengzhou University, Zhengzhou, Henan 450001, China; ^2^Department of Engineering Management, School of Transportation, Changsha University of Science and Technology, Changsha, Hunan 410114, China; ^3^Department of Engineering Management, School of Civil Engineering, Henan Polytechnic University, Jiaozuo, Henan 454001, China; ^4^Center of Excellence in Project Management, Department of Civil and Environmental Engineering, University of Maryland, College Park, MD, USA; ^5^Institute of Theoretical and Applied Informatics, Polish Academy of Sciences, Gliwice, Poland; ^6^Chaoyang University of Technology, Taichung, Taiwan

## Abstract

Building information modeling (BIM) is evolving as a digital infrastructure model for innovation in the construction field. The innovation-enabling potential of BIM has been highly neglected in the literature. This study explores the innovative potential of BIM, specifically its value in enabling construction innovation (CI). Through reflective research and a literature review, the relationship between BIM and CI is redefined, BIM-CI's value spectrum and underlying mechanisms are mapped and their required resources and activities are illustrated. The results indicate that different BIM applications provide various proinnovation environments wherein CI may flourish. Extra attention should be paid to BIM-enabled systematic collaborative innovation and digital innovation ecosystems with BIM as the core infrastructure that integrates the physical space with cyberspace to accelerate radical innovation. This study extends BIM management research by considering digital innovation and providing a new perspective for CI management theory and practice. The results will provide academics with a solid point of departure for developing relevant research and serve as a reference for practitioners who intend to utilize BIM for efficient innovation in construction projects.

## 1. Introduction

Since it was first proposed in the 1970s, building information modeling (BIM) has become the newest trend in the construction field. An effort has been devoted to pursuing the potential of BIM. Some have focused on the functionality provided by BIM (e.g., clash detection and energy analysis), while others have emphasized productivity and efficiency achievements enabled by BIM, such as existing construction management tools being integrated with open BIM to extend their capabilities in construction ecosystems [1] as well as integrating and enabling BIM capabilities to improve construction projects in combination with other innovations (e.g., new materials and new technologies such as three-dimensional (3D) printing, cloud computing, and robotics). These have led to advancements in the recognition and application of BIM.

However, regardless of the benefits related to productivity improvement in particular activities, the innovative capability of BIM has been highly neglected in the literature [2, 3]. Innovative capability involves the ability of BIM in enabling its user or organization/network to work differently (i.e., innovate) for improvement [2]. Evidently, construction innovation (CI) is pivotal to the ultimate success of construction projects and is key to the sustainable development of the construction sector [4]. Although the construction industry is often perceived as conservative, its inertia characteristics (e.g., stakeholder complexity, fragmentation, low profit margins, and low productivity rates) render it “ripe for digitization” [5, 6]. It has been demonstrated that due to the characteristics of digital technologies (i.e., convergence and reprogrammability), tremendous benefits are expected from digital technologies for CI. There are very few researchers who have noticed this aspect of the potential of BIM, and most relevant research has used case studies to describe the process or the outcome of CI enabled by BIM through the application of specific functionality (e.g., 3D representation) during certain stages (e.g., the design phase) of construction projects [2, 6]. Systematic research on the innovative capabilities of BIM is extremely scarce.

The essential reason for this lack of academic research and untapped practical potential may be the absence of a holistic picture of the value of the innovative capability of BIM in construction projects. Thus, the purpose of this conceptual study is to map a value spectrum of the ability of BIM to enable innovation in construction projects. To achieve this goal, reflective research and a qualitative literature review were conducted to reidentify the relationship between BIM and CI. By coupling CI classifications and BIM application modes, a value spectrum depicting a holistic picture of the innovative capability of BIM is mapped and analyzed, and its underlying mechanisms and required resources and activities are also illustrated.

Innovation-related research in the BIM management field mostly considers BIM as an innovative application or technology and examines its adoption, application, and implementation based on innovation diffusion theory or the technology acceptance model [3, 7]. A BIM application is an evolving, dynamic, and complex sociotechnical process. Indeed, BIM is more like an innovation engine rather than simply a technological innovation in the construction field. By exploring the innovative value potential of BIM and analyzing the value spectrum of innovations that enable BIM in construction projects, this study contributes to the body of knowledge by extending the scope of BIM management research considering digital innovation management. Furthermore, this study provides a new perspective for CI management theory and practice. Reshaping the relationship between BIM and CI and creating a value spectrum of the innovative capability of BIM will serve as a solid departure point for developing relevant research and guiding practitioners in executing project management based on BIM to develop innovative solutions in order to address engineering problems, improve efficiency, and build better projects.

## 2. CI in the Digital Era

The construction industry is a diverse, project-based sector [8]. Architecture, engineering, and construction (AEC) projects are distributed (i.e., designed and constructed by multiple, autonomous actors), heterogeneous (i.e., comprising communities with distinct skills, expertise, and interests), and sociotechnical (i.e., requiring trust, values, and norms as well as information technology (IT) capabilities and complex fabrication processes) [6]. The construction industry has always been regarded as a conservative economic sector because it involves large volumes of repetitive work. However, the completion of iconic mega projects, such as the Burj Khalifa Tower in Dubai and the Hong Kong-Zhuhai-Macao Bridge, also underscores the immense innovative potential of this sector.

Currently, the digitization of the construction industry is overwhelming. The inertia characteristics of the construction industry (e.g., stakeholder complexity, fragmentation, low profit margins, and low productivity) render it “ripe for digitization” [5, 9]. In the new digital era, the construction industry is required to build better buildings and offer better service in a shorter time and with tighter budgets, which pose more challenges to CI and make the improvement of its efficiency imperative [3]. Under such circumstances, digital technologies claim to be a promising new path for improving CI efficiency. Today's construction technology landscape offers a wide variety of innovative digital solutions for optimizing project constraints in terms of scope, time, cost, quality, and resources [5]. Based on the findings reported by the World Economic Forum regarding the likely impact of new technologies and global drivers influencing the future of construction, digitization-enabled innovation—which includes a range of capabilities such as data creation, management, reality capture, analytics, and automation control and tracking—is one of two broad technical trends [10]. The other trend is innovation in building materials, which is not included in the scope of this study [11].

Digital innovation involves the use of digital technology during the innovation process. Nambisan et al. [12] conceptualized digital innovation as the creation of, and the consequent change in, market offerings, business processes, or models resulting from the use of digital technology. Boland and Lyytinen [6] indicated that the two fundamental properties of digital technology are their reprogrammability and data homogenization. Together, they provide an environment of openness and flexibility that is used to create convergent and generative innovations [6]. By overviewing the evolutionary process of CI, Skibniewski and Zavadskas [13] indicated that advanced information and communication technologies develop rigidly and rapidly to ensure the realization of innovative solutions for emergent, dynamic, and complex engineering problems. BIM appears to be at the center of most advancements in digital construction [11]. After the implementation of BIM, a series of innovations, whether incremental advancements toward design and construction management or more radical advancements toward robotics or direct digital construction, will emerge and thus improve management efficiency [11]. Up until this point, BIM has been a prospective solution for improving the efficiency of CI [5].

### 2.1. Innovative Capability of BIM in Construction Projects

In the digital economic era, BIM is considered the main paradigm of the construction industry's technological transformation [14]. The BIM concept was originally proposed by Charles Eastman in the 1970s. Since then, issues related to BIM have attracted much attention. Research shows that innovation is one of the most popular topics in BIM management research [7].

Liu et al. [3] conducted a thorough bibliometric analysis of the BIM literature focused on innovation-related topics to investigate the latest status and trends. The results of the bibliometric analysis showed that the number of innovation-related articles in BIM research publications has increased over the past decade, while relevant research mostly depicted BIM as an innovative IT system and investigated its adoption, implementation, and performance based on innovation diffusion theory or the technology acceptance model from a technology-centered perspective. The characteristics of the ability of BIM to enable innovative action have generally been the focus of research. Innovative capability is the ability of technology to enable its users to pursue innovative activities [2]. Selçuk Çıdık et al. [2] highlighted that most relevant research still focused on what BIM technology can provide as a technological window of opportunity in construction projects. The topic of what and how people use BIM on a daily or routine operational basis to improve construction projects remains underresearched, which means that there is ambiguity regarding the innovative capability of BIM in construction projects. In other words, the ability of BIM to enable a construction project network to build or possess the ability to work differently (i.e., to innovate) in order to improve performance has been highly neglected. Thus, a clear illustration of the enabling capability of BIM for CI, that is, a clearly defined relationship between BIM and CI as well as a thorough analysis of the value level of the ability of BIM to enable CI, is highly necessary.

## 3. Methodology

Recently, there have been an increasing number of researchers claiming that divergent thinking and creative research methods are required for construction research [11]. In particular, conceptual advances are considered critical to the vitality of scientific research, which should be encouraged for prosperity [11, 15].

Research design and method selection are extremely effective and have the greatest potential for innovation when they match the nature of the research question [16]. In this study, the research question concerns the value spectrum of the ability of BIM in enabling CI. The purpose is to establish a conceptual or structural framework and detail, articulate, chart, describe, and depict the innovative capability of BIM. A conceptual study with a delineation goal can serve this research purpose [15].

Conceptual articles are devoted purely to thought-based conceptions and are devoid of data [15]. If inductive and deductive reasoning becomes difficult, and empirical data are either not available, are too costly for exploration, or are not particularly useful, then reflective research is a valid qualitative research method that is suitable for abductive topical reasoning and resolving this paper's research question [11]. Reflective research methodologies are frequently used in research groups; however, they are less often applied to academic research in the construction field. Nevertheless, Singh [11] claimed that this kind of exploratory research could benefit the research community by identifying outliers that are not limited by methodological rigor or statistical evidence [11]. In this research, the concept and characteristics of the innovative capability of BIM were perceived and constructed by thoroughly reviewing the relevant literature, including books, reports, and other sources. Given that CI enabled by BIM is a dynamically evolving, complex process, aside from literature reviews, authors have discussions with colleagues and attendees of international conferences to delineate the innovative value of BIM. Further, thought experiments have been utilized to map the value spectrum.

Actor network theory (ANT), path creation theory (PCT), trading zone theory (TZT), and digital innovation theory have been applied to assist the research process. Based on ANT, technology and other artifacts are regarded as actors shaping roles and relationships in networks [17]. Under this perspective, we can take BIM application in construction projects as a rearrangement of an innovation network. BIM, as the equivalent of other innovation actors, breaks the behavioral and interactional modes between innovation networks and provides a transparent and synchronizing information-sharing channel, thus cultivating propitious conditions for innovation to occur. Although the initial development of digital innovation theory in the context of an information system or the organizational science discipline is still in its infancy [12], the overwhelming development and application of pervasive digital technologies in various industries have challenged the underlying logic of traditional innovation theory. New logic for understanding the novel paradigm of innovation induced by pervasive digital technologies has been provided, for example, taking digital innovation management as a sporadic, parallel, and heterogeneous process of forking, merging, terminating, and refining problem-solution design pairs; shifts in participant cognition and sense-making in emerging distributed innovation as well as the importance of digital platforms with orchestration mechanisms [12, 18]. All the aforementioned examples provide a proper theoretical framework on which our reflective study may build. Regarding the driving mechanism under CI enabled by BIM, this study takes advantage of PCT and TZT to demonstrate how BIM stimulates innovation on the individual actor level and from the interaction perspective among multiple innovation network actors.

## 4. Redefining the Relationship between BIM and CI

Indeed, BIM is much more than a purely simple innovative technology; rather, it is an engine that promotes CI [19]. With the emergence of the digital economic era, BIM is considered the heart of smart/digital construction, and it will evolve as a digital infrastructure/platform for innovation in the construction field [9, 19]. Research has established BIM as a significant innovator [20]. The use of BIM can generate both technological and organizational innovation and enable potentially radical innovation that could disrupt the entire industry [9].

The current innovative capability of BIM has attracted the attention of researchers. For instance, Selçuk Çıdık et al. [2] proposed a conceptual continuum by synergizing the polarized functionalist (i.e., technology-centered) and nonfunctionalist (i.e., human-centered) perspectives on BIM to analyze its innovative capability. Boland and Lyytinen [6] found that BIM implementation in Frank O. Gehry's projects instigated diverse innovations, each of which created a wake of innovation. They concluded that Gehry's adoption of 3D BIM as the representational tool disturbed the ecology of interactions and stimulated innovations in his project networks by providing path-creating innovation trajectories in separate communities of practice, creating trading zones in which communities could create knowledge about diverse innovations, and offering a means for intercalating innovations across heterogeneous communities [6].

The aforementioned research concerning the innovative capabilities of BIM primarily focuses on the scope of design practice. Increasingly, the enabling effect of BIM on CI has been expanded to the project life cycle or beyond. In a deductive case study, Holmström et al. [19] investigated how sociotechnical actions such as adoption, reuse, and recombination of designs and processes empower the users of BIM tools to not only achieve productivity improvement in particular activities but also build system capabilities that enable new ways of working. Recently, the incorporation of BIM within the life cycle project management system in the construction field has been highlighted [21, 22]. All of the evidence previously shown demonstrates that the collaborative application of BIM throughout the entire life cycle of a construction project will disrupt the CI ecosystem and provoke the emergence of new innovation patterns, the reduction of communication costs, and the creation of digital convergence that may lead to new interactions and relationships between innovators. New knowledge, skills, and innovative possibilities, accompanied by the associated cognitive and social translation, can occur through the penetration of boundaries [23]. Therefore, by considering the life cycle project management theory and aligning it with the analytical framework used by Boland and Lyytinen [6], this study redefines the relationship between BIM and CI (Figure 1).

CI represents the engineering of problem-oriented innovation activities on the construction project level, which are usually completed collaboratively. The path for CI can be illustrated as a dynamic problem-solution matching process from both an individual organizational perspective (i.e., path creation) and a cross-organizational perspective (i.e., collaborative innovation). During these processes, the embeddedness of BIM serves to activate an individual organization's subjective initiative and accelerates collaboration between organizations to support CI.

A CI network enabled by BIM can be considered a digital ecosystem, a concept that Sawhney et al. [24] defined as a complex intermeshing of an interdependent group of organizations, people, products, and things that work on a shared digital platform for a mutually beneficial purpose and value creation. In this digital ecosystem, BIM, as a shared digital platform or orchestrator, as claimed by Nambisan et al. [12], offers a convergent approach to make project data available for multiple construction technology use cases (e.g., design management, document management process simulation, and project scheduling), thus becoming a key driver of innovation, emergent ecosystem behavior, and value creation [24, 25].

As demonstrated in Figure 1, BIM provides a window of opportunity for people to work differently to improve (i.e., innovate) on an operational level in separate practice communities [26]; path creation enabled by BIM provides innovation trajectories for actors within their organizational boundaries. For example, triggered by the demands and opportunities of high-profile projects and the state of development within each firm, participants in innovation networks enabled by BIM could mindfully invent their own innovation trajectories at different paces. Moreover, some could be more collaborative in their project organization, whereas others could be more experimental with materials and work practices [6].

According to Galison [27], when community boundaries cross or overlap during a project, a trading zone emerges. Owing to certain occasions or specific project tasks, various innovations can be interplayed in trading zones supported by BIM at permeable boundaries (shown in Figure 1 as the circles of dotted lines). In these trading zones, owners, designers, and contractors take artifacts (e.g., the BIM model) authorized by BIM as boundary objects or a common language to constantly refine and mutually adjust their interrelationship, thereby establishing a new interdependent network system so they can work together to produce innovative solutions for various design, construction, and delivery tasks. For example, based on a BIM platform, a construction company can work with trade contractors and third-party software developers to develop a tool for the real-time monitoring of construction workers to track worker safety, productivity, and well-being [24]. Path creation and the interplay of various innovations in trading zones will together lead to the so-called “wakes of innovation” enabled by BIM among the construction project network [6]. During these processes, knowledge evolves, learning occurs, and new action patterns are constructed.

Although BIM is an overall approach, BIM application is a dynamically evolving elaboration, because there are various functional specifications that can be implemented at different phases of a project's life cycle that can bring distinctive benefits and costs [26]. In reality, the application of BIM shows various possibilities with different functions (i.e., what BIM can do)—depending on when, where, and how people use it—and the interactions among individuals during its implementation (i.e., what people can do with BIM) [2]. Therefore, different types of BIM implementation will provide various levels of enabling effects on CI. However, people realize that BIM application has innovative value for construction projects and its users; however, the problem lies in how much value it brings and, particularly, how and in which situation the application of BIM can contribute to improving innovation efficiency for actors and networks of construction projects. This vagueness on the innovation value spectrum of BIM will consequently hinder construction projects in terms of taking full advantage of BIM to assist CI [26].

## 5. Value Spectrum of the Ability of BIM to Enable CI

### 5.1. Application Modes of BIM for Construction Projects

As previously mentioned, there are many possibilities of the application of BIM in construction projects, or various so-called “BIM application modes,” which are highly dependent on the type of interactions and relationships between the participants and how BIM is used [28]. Based on a case study of 25 BIM projects, Taylor and Bernstein [29] identified 4 BIM application modes—the visualization, coordination, analysis, and supply chain integration modes—which are consequently incrementally involved in the BIM experience. From the interoperability perspective, Grilo and Jardin-Goncalves [28] acknowledged that various interaction styles between project network actors can lead to different kinds of BIM utility, namely, communication, coordination, cooperation, collaboration, and channels. To sum up, because of the heterogeneous and systematic characteristics of BIM, BIM allows various application statuses to coexist in the construction industry. In this study, grounded on the aforementioned literature coupled with validation from senior BIM experts, the BIM application modes finally include the visualization, coordination, analysis, collaboration, and infrastructure modes.

### 5.2. Classification of CI

The classification of CI made by Slaughter has been commonly acknowledged in this field [8, 20], which will be applied to be the framework measuring the innovation value level of BIM in this study. As per changes regarding the concept and its linkage to other components, Slaughter classified CI into five clusters—incremental, modular, architectural, system, and radical—as shown in Figure 2.

According to Figure 2, incremental innovation is a small improvement to the standard practice based on existing experience and knowledge that influences the constraints of a specific element. Incremental innovation is usually more frequent in the construction industry than in other industries, such as the manufacturing industry. Actors from the entire value chain of a construction project can generate incremental innovation, for instance, by improving the products provided by a supplier or modifying the on-site construction process. Modular innovation is a relatively large change on the concept level within a component that has limited influence on the links to other elements or systems. The replacement of drawing with hands with computer-aided design (CAD) is a typical example of modular innovation, which only changes the way people design or draw in terms of the concept of design drawing; the changes to the relationships between design groups are very limited (i.e., they are still done using 2D paper drawings). Contrary to modular innovation, architectural innovation requires only trivial modification of concepts/elements but substantial revisions of the linkages with other elements/systems, such as incorporating self-compacting concrete. There is no obvious change to the concrete technique itself; it is the fact that under gravity, the fluidity, density, and homogeneity of concrete can be achieved without additional vibrating process changes in the interaction and interconnection between the activities related to this work. To achieve new functions or levels of performance, system innovation involves the integrative innovation of multiple innovations that requires the effective rearrangement of the subsystems comprising the system and relative changes in corresponding elements/systems. One example is the application of ballastless tracks in railway construction. The realization of systematic innovation, such as a ballastless track, requires the integration and coordination of multiple independent innovations (e.g., new orbital technology, new roadbed construction technology, and new maintenance technology). Radical innovation is a rare and unpredictable breakthrough in science or technology that might lead to the essential reform of an entire industry. For instance, the realization of the so-called digital twins (DT) mode may overturn the overall working logic for the construction industry.

The five types of innovation presented through the model can be arranged as per the scale of required change from the current state-of-the-art practice as an incremental, modular, architectural, system, and radical [4] (see Table 1).

The innovation classification system proposed by Slaughter [4] is utilized as the innovation value metric for measuring the innovative capability of BIM. On the one hand, the enabling effect of the application modes of BIM on CI is highly dependent on the willingness of actors in distinct communities (innovation path creation for concept change) and the interaction mode and interrelationship between various project network communities (linkage changes based on trading zones). On the other hand, assuming that innovation provides improvement through change, an innovation classification model based on the degree of change is appropriate. As demonstrated in Table 1, it is easier to describe the specific resources and activities (e.g., the timing of commitment, degree of coordination within the project team, need for special resources, and type and level of active supervision) [4] required for the application of BIM to enable the relevant level of CI. The alignment of the application of BIM with the classification of CI in exploring the value of the innovative capability of BIM is demonstrated in Table 1.

### 5.3. Analyzing the Value Level of BIM in Enabling CI

Based on the combination of Slaughter's [4] CI classification system and the BIM application mode summarized in this study (as shown in Table 1), the value spectrum for the innovative capability of BIM will be analyzed as follows (Figure 3). In Figure 3, the *x*-axis represents the evolution of BIM application modes, while the value of the innovative capability of BIM is demonstrated on the *y*-axis. As the scope and maturity level of a BIM application evolves, BIM application modes become more innovation-friendly environments. In other words, in different application modes, BIM provides different levels of innovation value. The wider the scope and the more mature the implementation of BIM, the higher the innovation value of its application in a construction project. Thus, the BIM application mode can be arranged according to the innovative value level of aspects such as visualization, coordination, analysis, collaboration, and infrastructure, as illustrated in Figure 3. This value proposition is not very solid and rigorous because incremental innovation to some actors may be considered modular or systematic innovation to other actors. Thus, the analysis and results herein are conducted on the construction project level and depart from the perspective of general project benefits.

#### 5.3.1. Visualization

Since the 1990s, the visualization mode of BIM has been widely applied in the construction industry, mainly for marketing or aesthetic requirements. The application of BIM visualization demonstrates a great effect on the design and construction phase. First, 3D models of BIM designed on the basis of a 3D entity component provided by suppliers highly improve the designing efficiency. Second, the application of BIM makes communication between designers and owners regarding design intentions more convenient, thus enabling effective information to be correctly conveyed to the relevant team member. In a virtual environment based on BIM, many kinds of “what ifs” can be demonstrated and compared intuitively, which can accelerate the optimization of design solutions by smoothing the communication and cooperation targeting design objectives and solutions. On the construction stage, compared to two-dimensional (2D) painting, 3D models enable contractors to more easily and clearly understand the owner's actual design requirements and intentions, which consequently reduces changes and requests for information subsequently in the project's life cycle.

The BIM visualization mode is essentially the transformation from 2D to 3D presentation technology. Therefore, the visualization mode of BIM application accelerates incremental innovation in construction projects at any time during the project. Incremental innovation enabled by BIM based on the visualization mode only involves small improvements and most of time is constrained by the scope of a single organization with no special resources or coordination required. The related supervision of the individual task level focuses on improving the notification manner and the supervisory competencies of the specific improved product, process, or service.

#### 5.3.2. Coordination

The coordination mode of BIM creates mutual benefits and avoids gaps and overlaps to connect various project activities and efficiently realize project objectives [28]. The coordination of the designing documents (e.g., structuring, plumbing, designing, and drawings) is an important example of this application mode. The coordination of complex systems is a common application in construction projects. The virtual 3D model is completed by various team members. No matter who the consultant is, a specialty manufacturer or a subcontractor, every team member will create their own model for their work purpose in a project. The general contractor will integrate these independent models to form a more holistic composite model that represents the overall picture of the project. Based on the coordination of the constituent components of the composite model, possible conflicts can be identified and resolved before execution; thus, this mode is also known as the conflict detection mode.

The coordination mode of BIM application invokes conceptual change of coordination issues in construction projects (e.g., design checks and clash detection) while having little influence on other systems. In this mode, innovative solutions are likely to be created in order to realize conceptual goals. Thus, the value level is in modular innovation. Modular innovations enabled by BIM are usually created during the design and bid stages. Because changes to the links to other components or systems are rare, very little explicit or implicit coordination within the project team is required. The resources required for a conceptual change must be prepared to conduct modular innovation enabled by BIM, such as the training required to install and maintain a component embodying a modular innovation. Relative supervisory activities (i.e., notification and review and technical competency) are required on the design and bid levels to ensure modular innovations enabled by BIM meet project objectives.

#### 5.3.3. Analysis

The analysis mode of BIM application realizes mutual benefits through sharing and cooperation. In the 3D virtual project environment based on BIM, the constructability and construction sequence can be clearly simulated. The entire arrangement of any specific task can be visualized in a 3D virtual environment based on BIM so that the schedule can be properly allocated. The BIM analysis mode provides the possibility to moderate and analyze construction costs and operations from the whole life cycle perspective. Moreover, BIM possesses many potential analytical capabilities for construction projects (e.g., energy consumption and lightning, wind flow patterns, and greenness). Theoretically, one central BIM model could be formed with all of the information needed by all contractors and consultants—information that contractors previously had to create independently from an architect's 2D blueprints [6]. The application of the analytical functionality of BIM requires construction project stakeholders to correctly and timely renew the information in the BIM model and share relevant information, which overturns adversarial relationships between project team workers and persuades them to constantly optimize project solutions from a holistic perspective. Indeed, the BIM analytical mode has not changed the way relevant analysis is done; however, it changes the interactions and links between different analysis systems: the data used for analysis can be retrieved if team workers correctly and timely input and share the BIM model information rather than repeatedly manually measure and calculate them.

In this BIM application mode, there is more potential for architectural innovation to occur, which requires the support and encouragement of organizations at the system level with strong management and control capabilities. For major changes to system or component links, architectural innovation enabled by BIM may require a greater degree of supervision and coordination among the affected parties. To ensure high-level performance from the completed system, the supervisory activities required include notification, agreement, and constant review and revision. Coordination among project team members based on BIM includes both official contract changes (e.g., if architectural innovations based on BIM lead to new project deliverables) and unofficial coordination (e.g., commitment to cooperate). Small conceptual changes may lead to a wide scope of BIM-enabled architectural innovations, from design-to-implementation, with special resources associated with complementary changes.

#### 5.3.4. Collaboration

The collaboration mode involves the full application of BIM in a construction project. Collaboration in a construction network based on BIM is a nonadversarial, team-based environment of mutual trust in which key participants are jointly involved in developing and augmenting the central BIM model throughout the life cycle of the project and where everyone understands and respects the input of others. The BIM model, as a central information resource, is a collaboration platform based on which the project's life-long activities are conducted (e.g., the owner develops an accurate understanding of the nature and needs of the project; the designer designs, develops, and analyzes the project; the contractor manages the construction of the project; the asset manager administers the operations of the project during the operation and decommissioning phase) [28, 30]. Through the collaborative application of BIM, the key participants jointly maximize the value of a construction project by mutually solving problems using proper contracts and fair risk/benefit sharing mechanisms. This application mode is pivotal to the formation and synergy of CI networks. The collaboration of a CI network based on BIM can bring about a synergistic effect that a single or a few functionalities or software programs cannot establish. The integrative application of BIM over the whole life cycle of a construction project provides reliable information and a knowledge-sharing platform for decision-making. Based on this, joint goals, joint responsibilities, and mutual understanding and respect are easily formed; team workers can communicate fluently and work together for innovative solutions rather than simply for efficient and similar results as in traditional approaches, thus creating a context for system innovation [3, 28]. With the execution of the collaboration BIM application mode, systematic CI has rich grounds to flourish upon.

Commitment to systematic innovation enabled by BIM is usually made during the conceptual design phase because it often involves new functions or increased levels of performance of an entity or a facility as a whole [4]. During the conceptual design phase, the collaborative innovation network enabled by BIM was designed, which facilitates the integration of a set of innovations. Coordination among network actors is assigned through official contracts or unofficial negotiations to reach a common sensibility of the information sharing and resources related to each innovation and their integration. The integrated project delivery method, or the design assistant kind of contract, is used by all project team members. The risk associated with system innovation may require active supervision by top engineering managers who are concerned with incorporating it into the project scope, obtaining agreements, and constantly reviewing its implementation and performance. These supervisors require technical and system competencies to assess the complementary changes needed to effectively implement the system innovation combined with organizational authority in order to ensure collaboration and integration. Professionals not only need to possess knowledge related to the individual innovation and its integration but must also master relevant collaboration knowledge concerning system innovations enabled by BIM [30].

#### 5.3.5. Infrastructure

With the coming digital economic era, the Internet 3.0 has enabled various possibilities for many different industries. In contrast to previous technological changes in the AEC industry, Morgan [9] claimed that the application of BIM has the potential to generate radical innovations that could disrupt the entire construction industry. The infrastructure application mode of BIM is more of a vision for the near future of the construction industry in the digitalized era wherein BIM is perceived as the most stable digital infrastructure [9, 19]. With BIM as the core digital infrastructure, the combination of divergent digital technologies (e.g., Internet of Things, 3D printing, and robotics) will thoroughly reform the productivity of the construction industry by welcoming the smart and digital construction era.

Radical innovation enabled by BIM entails not only financial and project risk but also the potential for technical failure, meaning that the commitment to this kind of innovation must be completed as early as possible, most often before the project is initiated (e.g., during the technical feasibility stage). Correspondingly, coordination of explicit and implicit cooperation and relative supervision requires the support of top management of all involved organizations. Consequently, the objective and scope of construction projects must be redefined, and the special resources required for radical innovation related to scientific or technological breakthroughs enabled by BIM might bring new challenges for top managers in terms of technical competencies in the specific scientific or technological area to monitor the implementation process and adjust the innovation activities accordingly [4].

## 6. Discussion and the Future BIM Agenda

Industry practitioners and academia mostly perceive BIM as a tool and an application and occasionally as a methodology. Consequently, research related to BIM mostly focuses on practice and application. BIM theory-building has been vastly limited [11]. Therefore, analogous to the development of management information systems as a discipline, Singh [11] claimed that there is a need to rethink the scope of BIM as a discipline emerging at the interface between construction, computer science, information management, and social science domains. The underpinning theoretical and conceptual questions regarding BIM have not been sufficiently investigated. Thus, our study joins this conversation by extending the BIM management research to the digital innovation management area by incorporating BIM into the domain of CI from a sociotechnical perspective [12]. In a CI network based on BIM, BIM may not only be an actor (i.e., a node) but also a relationship (i.e., a link) between elements or actors depending on the functionality used. This provides a new perspective for theory-building and practice of CI management. The underlying mechanisms for CI enabled by BIM will be analyzed based on path dependence theory and TZT in the following section. From the management information systems perspective, digital innovation and BIM-enabled digital innovation ecosystems will be utilized to describe the radical innovation value that BIM might be able to provide.

### 6.1. Mechanisms Underlying CI Enabled by BIM

As is depicted in Table 1, the enabling mechanism of incremental and modular innovation enabled by BIM based on the visualization and coordination modes is mainly path creation. The innovation trajectories of the involved actors are stimulated by the demands and opportunities of high-profile projects and the development status of each organization. Across the spectrum of engagement in path creation, actors may move at different temporal paces following their own logic and structure. The areas that incremental or modular innovation conduct are dependent on the professional identity and economic interests of the specific organization or community. Thus, they are sometimes more advanced in their use of technologies or are more experimental with their materials and work practices [6]. As the scope of change increases, the depth and width of the application of BIM in the analysis, collaboration, and platform modes rise. Aside from path creation, the innovating mechanism based on BIM focuses more on building trading zones. In these newly created interactive trading zones, the innovative level is aligned with the intensity of the interactions enabled by BIM. The infrastructure mode of the application of BIM leads to brand new innovation paths and disturbs the existing construction industry ecosystem, bringing new interaction modes among construction project-level innovation networks. As the establishment of trading zones becomes the dominant innovating mechanism, innovators of the CI network enabled by BIM gradually tend to innovate based on a shared identity, common vocabularies, and mutual understanding. In this situation, the innovation trajectories of separate actors or communities cross with those of others. Such interplay of innovations not only invokes new knowledge and skills for system innovation but also provide occasions for further upgrading of their separate innovation paths. To achieve higher value levels from innovation activities enabled by BIM, their tempo, structure, and logic should be aligned with a coherent and synchronized plan [6].

### 6.2. Systematic Innovation Enabled by BIM Based on Collaboration

The collaborative BIM application mode is the current goal of BIM implementation in a construction project. Collaborative BIM applications can reap value from incremental to system innovation, as shown in Figure 3. However, systematic innovation based on BIM through collaboration has not been thoroughly investigated in the literature [3].

BIM-CI is a dynamic problem-solution pairing process [12]. The implementation of BIM will change the interaction mode between the elements and actors involved and accelerate the formation and synergy between CI networks, thereby improving the innovative capabilities of BIM-CI networks [3]. BIM-CI networks are not designed but emerge from the interaction of individual social or technical elements or actors [31]. As an orchestrator, BIM plays the role of collaborative innovation platform, leading the innovation network to realize the synergistic effects of resource integration, effective communication, and common vision-building. The evolving and the emerging mechanism underlying this synergistic effect deserves further exploration.

Given the critical position of systematic innovation enabled by BIM in the value spectrum of the ability of BIM to enable innovation in construction projects, Liu et al. [3] proposed an inclusive systematic theoretical framework for collaborative CI enabled by BIM (also known as an “innovation pyramid”). This dynamic and evolving sociotechnical system contains six interdependent subsystems—contexts, actors, artifacts, processes, structures, and innovative tasks—as illustrated in Figure 4. In this system, actors possessing varying attitudes, requirements, and abilities use a range of technologies and tools (classified as artifacts) and work within a context with structures and a regulatory framework to take advantage of all of the resources (processes) to achieve the assigned innovative tasks [3].

To reach the synergistic effect of a BIM-CI network, the subsystems must fulfill enormous emerging requirements and overcome many challenges [32]. For example, new professional roles and skills are needed; when innovative new tasks (e.g., some construction companies have started to sell “Building as a Service”) for a new service emerge, the structure of the BIM-CI network (i.e., relationships and interrelationships, etc.) must be adjusted. Novel processes for the new form of business are required to implement workflow changes [33]. Further research should systematically examine the new problems faced by each subsystem. Additionally, the interactions, interrelations, and mutually adjusting effects of the subsystems on a macrolevel should also be investigated [3].

### 6.3. BIM as the Infrastructure for a Digital Innovation Ecosystem in Construction 4.0

Through collaboration, CI enabled focuses on reaping the systematic innovation value of BIM within the confines of a construction project. The extensive digitization of the construction industry persuades us to consider the bigger picture on an interproject and an industrial level and beyond.

Industry 4.0 has introduced digital technologies, sensor systems, intelligent machines, and smart materials to the construction industry [1]. This transformation is known as “Construction 4.0” [34]. With the adoption of advanced technologies, the processes and outcomes of CI have been gradually digitalized, thereby upending existing theories on innovation management by calling fundamental assumptions into question, such as the following: Are innovation boundaries definitional? Can innovation actors be predefined? Can innovation processes and outcomes be separated? [12].

Under such circumstances, the CI enabled by digital technologies urgently requires specific attention. The concept of digital innovation proposed in the information systems management field can be applied here. As explained by Khin and Ho [35], digital innovation is the development of new products, services, or solutions using digital technology (e.g., big data, Internet of Things, cloud computing, ontology, blockchain, data analytics, laser scanning, augmented and virtual reality, artificial intelligence, machine learning, and cyber-physical systems), in other words, in digital innovation, digital technologies and the associated digitizing processes form an inherent part of the new idea and its development, diffusion, or assimilation [12].

Digital innovation research brings digital technologies into the foreground of innovation management [31]. On the radical innovation value level, the DT mode is a revolutionary idea for realizing smart construction and Construction 4.0 [36, 37]. The key point for DT or Construction 4.0 is using BIM to connect virtual and actual building activities [35]. For the integration of this autonomous and synchronized cyber-physical system, BIM must collaborate with other cutting-edge Construction 4.0 technologies that embrace digital construction by transforming the construction industry into a dynamic environment [38].

To do so, a digital technologies ecosystem with BIM in the center as a common data infrastructure for enabling radical CI should be established. This “digital innovation ecosystem” refers to a dynamic, evolving network comprising heterogeneous elements [31]. The combined effects of several digital innovations in this ecosystem will bring about novel actors (and actor constellations), structures, practices, values, and beliefs that change, threaten, replace, or complement existing rules within organizations and fields [39]. How do we achieve an effective orchestration of these digital innovations? [12]. What is the structure of this complex, emerging, dynamic network? What are the emerging mechanisms underlying such digital innovation ecosystems? These are all equally significant issues that require examination. As digital technologies play an increasingly important role in construction and innovation activities, a challenging but fascinating set of security-related, ethical, legal, and regulatory issues also arise. How do we mitigate any potential negative influence while reaping the benefits of such digital technologies [40]? This is another research concern regarding digital innovation governance that should be investigated in future research.

## 7. Conclusions

This study explores a neglected area—the innovation-enabling potential of BIM in construction projects. Specifically, it analyzes and evaluates the value level of the ability of BIM to enable CI. The relationship between BIM and CI was redefined as shown in Figure 1. Besides the fact that BIM is often perceived as a typical construction innovation that offers efficiency and productivity improvements through its various functions or by extending BIM applications, BIM is instead an engine of CI. The main enabling mechanisms of BIM in terms of CI are path creation and trading zone building. Based on this fact, the value spectrum of the innovative capability of BIM was determined by coupling Slaughter's [4] CI classification system and BIM application modes in construction projects, as illustrated in Figure 3, with the resources and activities required to promote CI enabled by BIM. Additionally, the underlying innovating mechanisms are described in detail in Table 1. Various BIM applications provide different proinnovation environments wherein various levels of innovation may occur and flourish. The results indicate that extra attention should be paid to systematic innovation enabled by BIM based on collaboration and digital innovation ecosystems with BIM as their core infrastructure that integrates cyberspace and physical space to accelerate radical innovation.

Theoretically, this research extends the scope of the BIM management research considering digital innovation management issues and provides a new perspective for CI theory-building and management practice. The relationship between BIM and CI and the mapping of the value spectrum of the innovative capability of BIM provides researchers in this field with a novel perspective on the innovative capabilities of BIM. Relevant research should take the relationship structure and value spectrum map as departing points to design and develop further research. For practitioners, the detailed resources and activities required and the enabling mechanisms for relative levels of BIM-enabled CI can serve as good reference points to guide and inspire BIM-based project management practitioners to develop innovative solutions, solve corresponding engineering problems, improve efficiency, and build better projects.

However, regardless of its contributions, this study also has some limitations. This conceptual study is an initial exploration of the value spectrum of the innovative capability of BIM. Because the goal of this study is to conceptually delineate the innovative capability of BIM, the main research methods applied in this study were the literature review, reflective thinking, and thought experiments, during which abductive and logical reasoning was required, and traditional qualitative research methods (e.g., ground theory) were not utilized, which may cause some concern regarding the validity of the results. Thus, future qualitative and quantitative exploration of the value spectrum map of the innovative capability of BIM is required. In other words, these also create future opportunities to research BIM-enabled CI or digital innovation in the construction field. For instance, further research can apply more quantitative or mixed-methods research to validate the corresponding relationships between BIM and CI and develop relevant research questions, such as the following: Is there a corresponding relationship between the BIM application mode and the level of CI? Do the strategy and resources for enabling relative BIM-enabled innovation illustrated in this study suffice? Is the match between BIM and CI influenced by the delivery mode or owner involvement? How can the innovative capability of BIM in construction projects be activated?

As overwhelming as the development of Industry 4.0 was, the new concept of Industry 5.0 has also been recently proposed [41]. Industry 5.0 highlights the importance of human-centricity, sustainability, and resilience in addition to digitalization itself. Accordingly, the new paradigm of Construction 5.0, the construction industry's version of Industry 5.0, should be put on the agenda. As BIM plays a core role in this transformation, BIM/digital innovation-related research should pay extra attention to human-centered, environmentally friendly, and risk-related issues to promote the sustainable development of the construction industry.

## Figures and Tables

**Figure 1:** Relationship between BIM and CI.

**Figure 2:** The classification of CI adapted from Slaughter [4].

**Figure 3:** The value level of the innovative capability of BIM in construction projects.

**Figure 4:** Collaborative innovation enabled by BIM in construction projects by Liu et al. [3].

**Table 1:** Alignment of innovative capabilities of BIM with innovation models for construction adapted from Slaughter [4] and Murphy [20].

Type of CI	Definition	Scale of change	Example	Resource and activities required by BIM-enabled CI						Enabling mechanisms	BIM application mode
				Timing of commitment	Degree of coordination within the project team	Need for special resources	Supervision organizational level	Supervision type	Supervision competency		
Incremental	A small improvement to the standard practice based on existing experience and knowledge	Small	Modified construction process conducted on-site	At any time	None	None	At locus of improvement	Notification	Specific product or process	Path creation oriented	Visualization
Modular	A significant change in concept within a component but one that leaves the links to other components and systems unchanged		Computer-aided design (CAD)	At the design stage	None	For concept change	At design level	Notification, review	Technical competency		Coordination
Architectural	A small change within a component but a major change in the links to other components and systems		Self-compacting concrete	At the design-to-implementation stages	Among affected parties	For complementary changes	At the affected system level	Notification, agreement, review	System competency	Trading zone building oriented	Analysis
System	Multiple integrated innovations that complement each other to achieve new functions or levels of performance		Ballastless track	At the conceptual design stage	With all project team members	For integration of set of innovations	At top engineering management level	Project scope, agreement, review	Technical, system competency and organizational authority		Collaboration
Radical	A breakthrough in science or technology	Major	DT	At the technical feasibility stage	With top management from all involved organizations	For breakthrough	At top management level	Project objectives and scope	Specialized technical competency	Trading zone building + path creation oriented	Infrastructure

## Data Availability

No data were used to support this study.
